The article "Regenerative potentials of bone marrow mesenchymal stem cells derived exosomes or its combination with zinc in recovery of degenerated circumvallate papilla following surgical bilateral transection of glossopharyngeal nerve in rats" was retracted in 2025. Reasons: duplicated images; overlap with earlier publications; unreliable results or conclusions; concerns about the images.

# Regenerative potentials of bone marrow mesenchymal stem cells derived exosomes or its combination with zinc in recovery of degenerated circumvallate papilla following surgical bilateral transection of glossopharyngeal nerve in rats

**DOI:** 10.1186/s12903-024-05050-7

**Published:** 2024-10-30

**Authors:** Eman Mohamed Salem, Hamdy Rizk, Yara S. Abouelela, Abdelbary Prince, Adel Fathy Tohamy, Nawal A. Lasheen, Bassant A. Ezzat, Sana Mostafa

**Affiliations:** 1 Present Address: Oral Biology Department, College of Oral and Dental Surgery, Misr University for Science and Technology, Giza, 12568 Egypt; 2 Oral Biology Department, Faculty of Dentistry, Cairo University, Cairo, 115533 Egypt; 3 Anatomy and Embryology Department, Faculty of Veterinary Medicine, Cairo University, Giza, 12211 Egypt; 4 Department of Biochemistry and Molecular Biology, Faculty of Veterinary Medicine, Cairo University, Giza, 12211 Egypt; 5 Department of Toxicology and Forensic Medicine, Faculty of Veterinary Medicine, Cairo University, Giza, 12211 Egypt

**Keywords:** BM-MSC-derived exosomes, Glossopharyngeal nerve, Peripheral nerve injury, Circumvallate, Taste buds, Regeneration, Zinc chloride, Rats

## Abstract

**Background:**

Taste buds’ innervation is necessary to sustain their cell turnover, differentiated taste buds and nerve fibers in circumvallate papilla (CVP) disappear following glossopharyngeal nerve transection. Normally, taste buds recover to baseline number in about 70 days. Bone marrow stem cell (BM-MSC) derived exosomes or their combination with Zinc chloride are used to assess their potential to speed up the regeneration process of CVP following bilateral deafferentation.

**Methods:**

Twenty-eight male Sprague-Dawley rats were randomly divided into four groups; Group I: subjected to sham operation followed by IP injection of saline. The other experimental groups (II, III and IV) were subjected to surgical bilateral transection of glossopharyngeal nerve. Group II received single IP injection of saline. Group III received single IV injection of BM-MSC-derived exosomes (100 µg). Group IV received single IV injection of BM-MSC-derived exosomes and single IP injection of zinc chloride (5 mg/kg). After 28 days, CVP was dissected and prepared for histological and histomorphometric analysis, RT-PCR for cytokeratin 8 gene expression, ELISA to assess protein level of brain-derived neurotrophic factor, redox state analysis of malondialdehyde and glutathione content, followed by statistical analysis.

**Results:**

Histopathologically, group II exhibited great tissue damage with marked reduction in taste buds and signs of degeneration in the remaining ones. Group III was close to control group with marked improvement in taste buds’ number and structure. Group IV showed inferior results when compared to group III, with many immature taste buds and signs of degeneration. Statistical results showed that groups I and III have significantly higher values than groups II and IV regarding taste buds’ number, cytokeratin 8, and reduced glutathione. However, malondialdehyde demonstrated high significant values in group IV compared to groups I and III. Regarding brain-derived neurotrophic factor, group III had significantly higher values than group II.

The article "Regenerative potentials of bone marrow mesenchymal stem cells derived exosomes or its combination with zinc in recovery of degenerated circumvallate papilla following surgical bilateral transection of glossopharyngeal nerve in rats" was retracted in 2025. Reasons: duplicated images; overlap with earlier publications; unreliable results or conclusions; concerns about the images.

**Conclusion:**

BM-MSC-derived exosomes have superior regenerative potentials in acceleration of CVP and nerve healing following bilateral transection of glossopharyngeal nerve in contrary to its combination with zinc chloride.

**Graphical Abstract:**

**Supplementary Information:**

The online version contains supplementary material available at 10.1186/s12903-024-05050-7.

## Background

One of life’s greatest joys is the ability to enjoy different flavors. Loss of adequate gustatory function can lead to many difficulties, such as reduced appetite and altered eating patterns that potentially have an adverse impact on health [1]. Many different variables can cause taste changes or loss, including aging, trauma, chemical and drug exposure, smoking cigarettes, poor dental health, and malnutrition [2].

Taste perception from the posterior one-third of the tongue is conveyed mainly by circumvallate papillae (CVP), they receive bilateral innervation from the glossopharyngeal nerve (GPN) which convey multimodal sensations including taste, pain, tactile, and thermal signals [3]. CVP in rodents comprises a collection of intrinsic autonomic ganglionic neurons called the CVP ganglion. They are situated at the connective tissue core and play an essential role in events modulating taste transduction [4].

What makes the gustatory system special is the necessity to maintain taste buds’(TBs) innervation to sustain their cell turnover. It was reported that after GPN transection, TBs, and nerve fibers completely disappeared after a few days post-surgery in rats [5, 6].

Remarkably, taste-related nerve injury may have serious and enduring effects. GPN is highly susceptible to environmental insults caused by commonplace events such as falls, mishaps at work and sports, as well as more critical ones like motorbike or car accidents [7–9]. Moreover, GPN is at risk of surgical transection, this mostly is due to its route along the palatine tonsil which makes it more vulnerable to injury during tonsillectomy. Treatment for sleep apnea and surgery on the skull base pose additional surgical hazards [10].

The article "Regenerative potentials of bone marrow mesenchymal stem cells derived exosomes or its combination with zinc in recovery of degenerated circumvallate papilla following surgical bilateral transection of glossopharyngeal nerve in rats" was retracted in 2025. Reasons: duplicated images; overlap with earlier publications; unreliable results or conclusions; concerns about the images.

Peripheral nerve (PN) injuries heal quite slowly, and the effectiveness of current therapies is still relatively low. There are several techniques to enhance axonal regeneration and reinnervation of target organs depending on the kind and extent of nerve damage, including surgical and non-surgical treatment procedures [11, 12]. These strategies like autologous nerve grafting and nerve guide conduits offer some degree of axon regeneration although the recovery level is still scarce, highlighting the need for more effective treatment [13].

Bone marrow mesenchymal stem cells derived exosomes (BM-MSC) are a subclass of extracellular vesicles synthesized by stem cells and involved in different intercellular communication. These bio-nanoparticles include lipids, proteins, and nucleic acids as their natural payload [14, 15]. They reveal outstanding clinical applications, such as treatment modalities, drug delivery, and tissue regeneration [16].

Several previous in-vitro studies proved the ability of BM-MSC-derived exosomes for promoting nerve healing. BM-MSC-derived exosomes can inhibit neuroinflammation and promote healing of nerve damage by preventing the proinflammatory cytokines expression and increasing the anti-inflammatory cytokines in-vitro [17]. Furthermore, BM-MSC-derived exosomes promoted peripheral nerve regeneration in the dorsal root ganglion neurons model [18, 19].

The therapeutic possibilities of exosomes in neurodegenerative disabilities are seemingly promising. Several studies confirm that they are an encouraging treatment option for enhancing axonal regeneration following PN injuries [20, 21]. However, the clinical translation of exosome treatments is still confronted with issues related to the exosome origin, dose, and targeted delivery [13].

Zinc (Zn^2+^) micronutrient is crucial for many metabolic processes as it can catalyze over 100 enzymatic reactions in the body. It controls the proliferation, survival, and differentiation of neurons at various phases of neurogenesis [21]. After nerve injury, Zn^2+^ supplementation was proven to enhance myelination, axonal regeneration, neuronal survival, and reinnervation of target organs [22]. Moreover, Zn^2+^ is considered part of the cell-tissue antioxidant defense network [23].

According to the pervious mentioned data, the present study was conducted to examine the regenerative potentials of BM-MSC derived exosomes alone or its combination with Zn^2+^ as a co-treatment in recovery of degenerated CVP following surgical bilateral transection of GPN in rats.

## Materials and methods

### BM-MSC isolation & culture

Three male Sprague Dawley rats (6-week-old, weighing 100 ± 20 g). Rats were anesthetized with Diethyl ether and were euthanized by decapitation in a laminar flow cabinet sterilized with 70% (v/v) alcohol. The skin of both legs was removed and then gently remove the tissue, fat, and muscles surrounding the tibia and femur to expose the bone. The isolated bones were transferred into a sterile 6-cm Petri dish filled with 6 mL of cold phosphate-buffered saline (PBS). Both extremities of the tibiae and femora were cut. The bones were flushed by 2-mL Dulbecco’s Modified Eagle Medium (DMEM) [Gibco-BRL, Gaithersburg, USA] (low glucose with stable glutamine, 10% fetal bovine serum (FBS), 1% antibiotic mix (penicillin-streptomycin), then transferred into a sterile 15 ml Falcon® tube. The isolated Bone marrow solution was cultured into sterile flasks containing DMEM (high glucose with stable glutamine, 10% FBS, 1% antibiotic mix) in an incubator, at 37 °C in a humidified atmosphere (5% CO_2_). The media changed after 24 h to remove nonspecific cells, then it changed every three days until cells reached 80–90% confluency.

The article "Regenerative potentials of bone marrow mesenchymal stem cells derived exosomes or its combination with zinc in recovery of degenerated circumvallate papilla following surgical bilateral transection of glossopharyngeal nerve in rats" was retracted in 2025. Reasons: duplicated images; overlap with earlier publications; unreliable results or conclusions; concerns about the images.

### (BM-MSC) derived exosomes isolation & purification

Exosomes were prepared in NAWAH Scientific Lab, Cairo, Egypt. Briefly, Mesenchymal stem cells were cultured till the third passage with 70–90% confluency. The complete media was changed, and the flasks were washed twice using PBS.

Cells were left in media without serum (low glucose DMEM with 1% Antibiotic mix) and incubated in 5% CO_2_ at 37 °C to produce exosomes for two days. After 2 days, the media containing exosomes were collected, centrifugated (2500 rpm for 10 min) to get rid of any cells, and filtered using 0.45 μm then 0.22 μm filter to remove any debris and take the supernatant. This was followed by Ultracentrifugation [Beckman Coulter OptimaTM L-80XP 100,000 g avg at 4 °C for 90 min with a Type 50.2 Ti rotor (k-factor: 157.7)] to pellet exosomes.

After cautiously discarding the supernatant, crude exosome-containing pellets were once again mixed in 1 milliliter of ice-cold PBS and collected. Following another round of ultracentrifugation, the exosome pellet was resuspended [24]. Following the manufacturer’s instructions, the concentration of exosomes was determined using the bicinchoninic acid protein assay kit (Novagen). Reagents were employed at a 2:100 ratio, with 4% cupric saltate and bicinchoninic acid solution.

### (BM-MSC) derived exosomes characterization

Purified BM-MSC derived exosomes were recognized using transmission electron microscopy, where it showed a typical cup-like morphology, their vesicular morphology was circular, intact and the size range did not exceed 120 nm (Fig. 1A). The average size of exosomes was analyzed using the Malvern Zetasizer Series (Fig. 1B).

The article "Regenerative potentials of bone marrow mesenchymal stem cells derived exosomes or its combination with zinc in recovery of degenerated circumvallate papilla following surgical bilateral transection of glossopharyngeal nerve in rats" was retracted in 2025. Reasons: duplicated images; overlap with earlier publications; unreliable results or conclusions; concerns about the images.

The exosomes identification was established by Flow cytometric analysis (Beckman Coulter®, USA) as the exosomes expressed CD90, CD73, CD9 and CD63 surface markers. The exosomes resuspended in a mixture of PBS and 3% fetal bovine serum containing saturating concentrations (1: 100) dilution of the following fluorescein isothiocyanate-conjugated anti-human monoclonal antibodies: anti CD90, anti-CD73, anti CD9 and anti-CD63 (BD Pharmingen). Samples were tested using forward scatter analysis (Becton-Dickinson, Canada) (Fig. 1C).

**Fig. 1:** BM-MSCs derived exosomes characterization. **A** Exosomes structure by transmission electron microscopy; **B** Particle size analysis **C** Flowcytometric analysis of CD73, CD90, CD9 and CD63

### Zinc chloride preparation

ZnCl_2_ hydrate chemical (98% pure, solid) was obtained from (Gomhorya company, Egypt). ZnCl_2_ dose was calculated and dissolved in deionized water then administered in a plastic syringe (1 ml), as a single IP dose of 5 mg/kg [25].

#### Animal study approval number

The current work was conducted under the permission of the Institutional Animal Care and Use Committee (IACUC), Cairo University (Approval number: III F 31 22). This research was carried out following the ARRIVE guidelines and regulations (https://arriveguidelines.org*).*

### Sample size

The sample size was calculated according to the St. John’s et al. study [26].

A minimum number of animals (6 per group) will be sufficient for good statistical analysis. With concern to about 20% mortality rate due to the surgery, a total sample of 28 rats (7 per group) was used to detect an effect size of 0.4, a power of 0.8, a two-sided hypothesis test, and a significance level of 0.05. Calculations were completed using the G*power program (version:3.1.9.7, Germany).

### Animals

Twenty-eight healthy male Sprague Dawley rats with weights ranged 150–200 g were purchased from the animal house of Misr University for Science and Technology, Giza, Egypt. Rats were housed in an enriched environment with controlled room temperature 25 ± 2 °C and 12/12 h light/dark cycle. They had access to a normal diet and water with one week acclimatization period before surgery. Rats were housed in polypropylene cages with 48.5 cm length× 33 cm width × 21 cm height (Al-Alamia Company, Giza, Egypt). After surgery, all rats were housed separately till complete healing then placed as three or four per cage.

The rats’ welfare was reported by the attending veterinarian who managed any recorded pain or distress according to the ethical protocols for animal handling that were supervised by the animal facility at Misr University for Science and Technology.

The article "Regenerative potentials of bone marrow mesenchymal stem cells derived exosomes or its combination with zinc in recovery of degenerated circumvallate papilla following surgical bilateral transection of glossopharyngeal nerve in rats" was retracted in 2025. Reasons: duplicated images; overlap with earlier publications; unreliable results or conclusions; concerns about the images.

#### Animals grouping

The Random Sequence Generator tool (randomizer.org) was used to randomly distribute the rats into four groups (one control and 3 experimental) each incorporating 7 rats as shown in Table 1. Rats were matched blindly with the numbers (from 1 to 28) by the attendant technician, then they were assigned in their groups following the program suggestions.

A sham operation was performed on the rats of group I (negative control), followed by an intraperitoneal (IP) injection of 0.9% saline. Experimental groups were subjected to surgery in which the GPN was transected bilaterally. Group II (positive control) received an IP injection of 0.9% saline post-surgery. Group III received a single dose of 100 µg BM-MSC-derived exosomes intravenously (IV) through the tail vein [27]. Group IV received a single dose of 100 µg BM-MSC derived exosomes and a single IP injection of 5 mg/kg of zinc chloride (ZnCl_2_) [25].

**Table 1:** Animal grouping and study design

Group	Rats’ no.		Intervention	Injection
I	7		Sham operation	Saline IP
II	7		Bilateral cutting of glossopharyngeal nerve	Saline IP
III	7		Bilateral cutting of glossopharyngeal nerve	Exosomes IV
IV	7		Bilateral cutting of glossopharyngeal nerve	Exosomes IV + ZnCl_2_ IP

#### Surgery procedure

Rats were anesthetized by a mixture of ketamine 40–100 mg/kg IP /xylazine 5–13 mg/kg IP [28]. Rats were manipulated with back recumbency then hair clapped in its ventral head region. A midline incision in the skin was applied, followed by blunt dissection using Metzenbaum scissors (Curved 6” Surgical Veterinary Stainless Steel, Premium Instrument Company, US) to reflect subcutaneous fascia, with reflection of the submandibular and sublingual glands [6]. Group I was sutured after this step (sham operation) while other experimental groups were subjected to bilateral transection of GPN. GPN was visualized at the medial face of the caudal belly of the digastric muscle and held by an Instrapac® micro forceps No. 7 [26], then the nerve transacted with micro scissors on both sides. Fascia and skin were sutured by Vicryl 6/0 suture material with an antiseptic solution on the suture to avoid infection. All steps were applied bilaterally, rats of group I received the same procedure but without transection of GPN (Supplementary Fig. 1A).

Antibiotic was administrated for 3 days following surgery to prevent infection, each rat received (vancomycin15 mg/kg IV, Mylan N.V., Pennsylvania, USA) for 3 days [29]. Analgesics (5 mg/kg I.M of Ketoprofen, Anafen®; Merial-Canada) were supplied once daily for 3 days post-surgery or when pain was monitored [30]. At the end of 28 days, rats of all groups were euthanized with an overdose of sodium thiopental 80 mg/kg IV (Anapental 1, P2-55-011, Sigma Tec Pharma–Egypt) [31]. Once the animals were anaesthetized, confirmation of death was carried out by physical method (decapitation). The heads were dissected, and the tongues were collected for examination.

The article "Regenerative potentials of bone marrow mesenchymal stem cells derived exosomes or its combination with zinc in recovery of degenerated circumvallate papilla following surgical bilateral transection of glossopharyngeal nerve in rats" was retracted in 2025. Reasons: duplicated images; overlap with earlier publications; unreliable results or conclusions; concerns about the images.

After 28 days, CVP was dissected from the tongues of all rats and prepared for histological and Histomorphometric analysis, RT-PCR for cytokeratin 8 gene expression, ELISA to assess protein level of brain-derived neurotrophic factor, redox state analysis of malondialdehyde and glutathione content, followed by statistical analysis.

### Histopathological examination and histomorphometric analysis

CVP was dissected out from the tongues, placed in a plain vacutainer (Voma Med® 5 ml, Turkey) and immediately fixed by immersing in 10% neutral buffered formalin solution for 48 h. The samples were dehydrated in ascending grades of ethanol, cleared in xylol, and embedded in paraffin wax according to standard protocol [32].

Serial coronal sections were cut (7 mm-thick) using a microtome (LEICA RM2255, Leica Biosystems, Nussloch GmbH) and stained with H&E (Sigma®, St. Louis, MO, USA) for histological and morphometric analysis using Leica DM300 light microscopic (Leica Microsystems, Inc., Switzerland).

TBs count in each papilla was determined according to Pai et al., 2007. In each sample, twenty TBs were marked randomly, and the number of sections needed for each TB to appear was documented. This average was then divided by the total number of TB sections to calculate the total TB count [33]. Each section was examined with a magnification of x40, and the Image J (Version:1.53t) computer system was used to calculate the TBs after marking them with green crosses.

### Reverse transcription polymerase chain reaction (RT-PCR)

RT-PCR was carried out to obtain a relative measure to the amount of cytokeratin 8 (CK8) gene expression in the whole CVP. According to the manufacturer’s instructions, total RNA was extracted using the easy-spin total RNA Extraction Kit (iNtRON Biotechnology DR, Cat. No. 17221) according to manufacturers’ instructions. The quantity and quality of RNA were evaluated using a Nanodrop ND-1000 spectrophotometer (Nanodrop Technologies).

For quantitative expression of CK8 target gene, 5 µL of the total RNA from each sample was used for cDNA synthesis by reverse transcription, the cDNA was produced using MMuLV Reverse Transcriptase (NEB#M0253). The cDNA was amplified utilizing the HERAPLUS SYBR Green qPCR Master Kit (#: WF10308002). QuantStudio™ 5 Real-Time PCR System, 96-well, 0.2 mL, (ABI#A28139) was operated as follows: 95 °C for 2 min for enzyme activation followed by 40 cycles of 10 s at 95°C, and 30 s at 60 °C. The internal control used was GAPDH gene, and results were assessed by the ΔΔCt method. The data was analyzed using data analysis software, Version 1.4.5.

The article "Regenerative potentials of bone marrow mesenchymal stem cells derived exosomes or its combination with zinc in recovery of degenerated circumvallate papilla following surgical bilateral transection of glossopharyngeal nerve in rats" was retracted in 2025. Reasons: duplicated images; overlap with earlier publications; unreliable results or conclusions; concerns about the images.

The primer sequences specific for each gene are demonstrated in Table 2 [34].

**Table 2:** Primer’s sequence

Target gene	Primer sequence
Cytokeratin 8	Forward 5’ TTG AAA CCC GAG ATG GGA AA 3’ Reverse 5’ GGC CAT TCA CTT GGA CAT GAT 3’
GAPDH	Forward 5’ GGTCATCCCAGAGCTGAACG 3’ Reverse 5’ TCAGTGTTGGGGGCTGAGTT 3’

### Biochemical analysis

The samples of CVP were prepared by rinsing tissues with phosphate-buffered saline (PBS) to remove excess blood, and placing it in iced PBS, then freezing at -80˚C. The frozen samples were chopped into small parts and homogenized in 5 ml cold buffer (0.5 g of Disodium phosphate added to 0.7 g of Monosodium phosphate dissolved in 500 µl deionized water, pH = 7.4). Then the homogenates were centrifuged at 4000 rpm for 15 min at 4˚C, and the supernatant was collected for Enzyme Linked Immunosorbent Assay (ELISA) and redox state analysis.

The protein level of Brain-derived neurotrophic factor (BDNF) was measured in the tissue supernatants using a commercially available ELISA kit (Cusabio Technology LLC, USA), according to the manufacturer’s instructions.

Commercially available kits were used to assess the CVP content of malondialdehyde (MDA; Colorimetric Method, Cat. No. MD 25 29; Biodiagnostic, Egypt) and reduced glutathione (GSH; Colorimetric Method, Cat. No. GR 25 11; Biodiagnostic, Egypt) following the kit instructions.

#### Statistical analysis

Numerical data were presented as mean with 95% confidence intervals (CI), standard deviation (SD), minimum (min.), and maximum (max.) values. They were tested for normality and variance homogeneity by viewing distribution and using Shapiro-Wilk’s and Levene’s tests, respectively. They were found to be normally distributed with homogenous variances across groups and were tested using one-way ANOVA followed by Tukey’s post hoc test. Correlation analyses were made using Spearman’s rank-order correlation coefficient. The significance level was set at *p* < 0.05 within all tests. Statistical analysis was performed with R statistical analysis software version 4.4.0 for Windows [35].

## Results

### Histopathological results

The histopathological examination of group I showed a normal CVP appearance with a narrow base and broad surface surrounded by two deep troughs. The papilla was covered by stratified squamous epithelium with a thin keratin layer, the gustatory epithelium comprised numerous barrel-shaped TBs filling the whole epithelial thickness at both trough sides with taste pore opening into the troughs (Fig. 2A, B). The central core of connective tissue (CT) consisted of mature collagen bundles, spindle-shaped fibroblasts and small blood vessels with few inflammatory cells. At the core of the papilla, a dense ganglionic plexus (CVP ganglion) covered by a dense connective tissue capsule was located. The ganglion contained several large, rounded ganglion cells with eccentric deeply stained nuclei and basophilic cytoplasm (Fig. 2A, C).

The article "Regenerative potentials of bone marrow mesenchymal stem cells derived exosomes or its combination with zinc in recovery of degenerated circumvallate papilla following surgical bilateral transection of glossopharyngeal nerve in rats" was retracted in 2025. Reasons: duplicated images; overlap with earlier publications; unreliable results or conclusions; concerns about the images.

Group II showed obvious outline deformity, the epithelium appeared thinner in thickness and the troughs were obviously narrower and shorter compared with the control group. TBs were notably decreased in number (with some areas of gustatory epithelium devoid of TBs) and they were swollen with signs of taste cells’ separation or degeneration (Fig. 2D, E). The CT core showed areas of collagen fibers degeneration and separation. The ganglion cells exhibited degenerations’ signs including reduced size, pyknotic nucleus and darkly stained cytoplasm. Focal aggregation of marked inflammatory cells infiltrate was also evident (Fig. 2D, F).

Group III showed a papilla outline closer to normal, the covering epithelium was thinner in thickness, with deep narrow troughs which were slightly straighter than normal. TBs were numerous and normal in shape and number (Fig. 3A, B). Dense CVP ganglion was located at the CT core and covered by a dense connective tissue capsule with several normal-shaped ganglionic cells. The CT core has few inflammatory cells (Fig. 3A, C). Surgical results is presented in (Supplementary file 1 Fig. 1B).

Group IV showed slight deformity of the general outline. The gustatory epithelium increased in thickness with a noticeable rise in immature TBs’ number that arranged in different levels, while some of them showed signs of degeneration (Fig. 3D, E). The ganglion nerve plexus was smaller in size with signs of ganglion cells degeneration. Areas of collagen fibers degeneration and disorientation were detected with focal infiltration of inflammatory cells (Fig. 3D, F). Surgical results is presented in (Supplementary file 1 Fig. 1).

**Fig. 2:** Photomicrograph of CVP showing; **Group I: A** Normal papilla appearance where it is covered with normal keratinized epithelium (Ep), surrounded by two deep narrow troughs (arrows), gustatory epithelium filled with numerous taste buds (T), and connective tissue core (CT) **(H&E**,** 100x). B** Gustatory epithelium with normal shaped taste buds and taste pores (short black arrows), undulated bundles of subgemmal nerve fibers supplying taste buds (red arrows), and blood vessel (b.v) **(H&E**,** 400x). C** Ganglionic nerve plexus surrounded by connective tissue capsule (arrowheads) **(H&E**,** 400x). Inset**: Higher magnification showing normal shaped ganglion cell (pointed arrow), and prominent Schwann cells nuclei (curved arrows) within nerve plexus **(H&E**,** 1000x). Group II: D** Deformed outline of papilla where it is covered with thinner epithelium and detached keratin layer (Ep), surrounded by short narrow troughs (arrows) gustatory epithelium were nearly devoid of taste buds except for few degenerated ones (T), and focal aggregation of inflammatory cells (F) **(H&E**,** 100x). E** Swollen taste buds with signs of cell degeneration and separation (short black arrows), and few isolated subgemmal nerve fibers (red arrows) **(H&E**,** 400x). F** Remnants of degenerated ganglion tissue (arrowheads), disoriented collagen fibers (asterisk) and a marked increase in inflammatory cells infiltration (F) **(H&E**,** 400x). Inset**: Higher magnification showing shrunken degenerated ganglion cells with darkly stained nuclei (pointed arrows) and darkly stained Schwann cells nuclei (curved arrows) **(H&E**,** 1000x)**. (Original uncropped images are provided in the supplementary file 2 Figs. 4–7)

**Fig. 3:** Photomicrograph of CVP showing; **Group III: A** The CVP covered with thin keratinized epithelium (Ep), it is surrounded by two deep narrow and straight troughs (arrows), gustatory epithelium comprises normal taste buds (T), connective tissue core infiltrated with inflammatory cells (F) **(H&E**,** 100x). B** Normal taste buds with taste pores (short black arrows), and bundles of subgemmal nerve fibers supplying taste buds (red arrows) **(H&E**,** 400x). C** Normal CVP ganglion surrounded by dense CT capsule (arrowheads) **(H&E**,** 400x). Inset**: Higher magnification showing normal shaped ganglion cells (pointed arrows) within nerve plexus **(H&E**,** 1000x). Group IV: D** slight deformity in the CVP outline with thinner covering epithelium, it is surrounded by deep wide troughs that reflect outward (arrows), gustatory epithelium with multiple immature taste buds that arranged in different levels, some of them showed signs of degeneration (T), and inflammatory cells infiltration in connective tissue (F) **(H&E**,** 100x)**. **E** Multiple swollen taste buds with signs of degeneration (short black arrows), few disoriented subgemmal nerve fibers (red arrows) **(H&E**,** 400x). F** Degenerated ganglion cell within shrunken nerve plexus (arrowhead), collection of Schwann cells with darkly stained nuclei (curved arrows) **(H&E**,** 400x). Inset**: Higher magnification showing shrunken ganglion cells with darkly stained nuclei (pointed arrow) **(H&E**,** 1000x)**. (Original uncropped images are provided in the supplementary file 2 Figs. 4–7)

The article "Regenerative potentials of bone marrow mesenchymal stem cells derived exosomes or its combination with zinc in recovery of degenerated circumvallate papilla following surgical bilateral transection of glossopharyngeal nerve in rats" was retracted in 2025. Reasons: duplicated images; overlap with earlier publications; unreliable results or conclusions; concerns about the images.

### Statistical results

The results of intergroup comparisons are presented in Table 3. Results demonstrated that for all parameters there was a significant difference between tested groups. For the number of TBs, CK8, and GSH, post hoc pairwise comparisons verified that groups (I) and (III) have significantly higher values than groups (II) and (IV). For MDA, the results exhibited that group (IV) has significantly higher values than groups (I) and (III). In addition, group (II) has significantly higher values than group (I). For BDNF, the results revealed that group (I) has significantly higher values than other groups. Moreover, group (III) has significantly higher values than group (II). The correlations between different variables are presented in Table 4. Results showed that there were strong negative correlations between [GSH and MDA], [MDA and BDNF], [MDA and CK8], and [MDA and TBs’ number]. Other correlations were strong and positive. Mean and standard deviation values for different measurements are presented in (Supplementary file 1 Figs. 2 and 3).

**Table 3:** Intergroup comparison

Measurement	(Mean ± SD)				f-value	*p*-value
	Group (I)	Group (II)	Group (III)	Group (IV)		
GSH (mg/g)	25.15 ± 5.01^A^	10.75 ± 2.66^B^	21.71 ± 5.06^A^	8.35 ± 1.50^B^	**13.41**	0.002*
MDA (nmol/g)	21.94 ± 6.24^C^	45.43 ± 5.70^AB^	30.60 ± 5.42^BC^	51.45 ± 6.16^A^	**15.78**	0.001*
BDNF (pg/mg)	162.00 ± 4.58^A^	121.67 ± 2.52^C^	141.00 ± 4.00^B^	132.67 ± 5.69^BC^	**46.16**	< 0.001*
Relative Quantity of CK8 mRNA	0.97 ± 0.06^A^	0.16 ± 0.05^B^	0.96 ± 0.04^A^	0.20 ± 0.03^B^	**320.60**	< 0.001*
Taste buds’ number per papilla	16.80 ± 2.31^A^	4.27 ± 0.31^B^	15.20 ± 2.27^A^	5.60 ± 1.31^B^	**40.56**	< 0.001*

Values with **different superscripts** within the **same horizontal row** are significantly different, *significat at (*p* < 0.0)

**Table 4:** Correlation matrix

Variables	Correlation coefficient				
	GSH	MDA	BDNF	CK8	TBs
TBs	0.643*	-0.804*	0.769*	0.789*	
CK8	0.683*	-0.648*	0.859*		0.789*
BDNF	0.664*	-0.713*		0.859*	0.769*
GSH		-0.804*	0.664*	0.683*	0.643*
MDA	-0.804*		-0.713*	-0.648*	-0.804*

*Significant at (*p* < 0.05)

## Discussion

PN regeneration is one of the most challenging treatment strategies after neural injury, one of the main obstacles is the slow rate of axon growth (about 1 mm daily). Even though PN can regenerate on its own, in many situations it is inhibited by the length of time that passes between an injury and treatment. Scar development may impede or severely limit self-regeneration. Therefore, it’s important to create cutting-edge therapeutic approaches to speed up the regeneration process [13, 37].

The article "Regenerative potentials of bone marrow mesenchymal stem cells derived exosomes or its combination with zinc in recovery of degenerated circumvallate papilla following surgical bilateral transection of glossopharyngeal nerve in rats" was retracted in 2025. Reasons: duplicated images; overlap with earlier publications; unreliable results or conclusions; concerns about the images.

The peripheral gustatory system of rats is an interesting model to test neural variations due to its remarkable plasticity and robust regeneration. Rats’ neuronal anatomy and taste pathway are similar to humans, and severe GPN injury leads to a dramatic loss of TBs [38, 39].

It was confirmed from previous studies in rats that following GPN transection, the number of TBs in CVP recovered to 80% of the normal level in about 70 days. The first reappearance of TBs in CVP after denervation was found to be within 17 to 28 days [26, 36, 37]. Thus, the time course of the current work was chosen to be 28 days (to be closer to the first appearance date), to assess if the experimented materials will accelerate the regeneration process and to ensure that TBs did not fully regenerate after denervation.

Those findings agreed with the histopathological and histomorphometric results of the ongoing study that exhibited utmost damage in group II (positive control) in response to GPN transection, and TBs notably decreased in number with signs of degeneration. It was proven that gustatory nerve sectioning in mice causes apoptosis of TB cells, which diminished in size and number after an average of one week, while completely disappearing at 11 days [38].

The extensive destruction of nerve cells and focal aggregation of inflammatory cells at the site of CVP ganglion in the ongoing study was explained by the significant neutrophil and macrophage infiltration at the location of the nerve damage in experimental models of neuropathy. Additionally, both Schwann cells (SCs) and cytotoxic T lymphocytes activate and attract nearby phagocytes to the site of injury to phagocytose the myelin and engulf synaptic connections leading to the degeneration of neurons. Moreover, they release cytokines and neurotrophic factors that direct the subsequent regeneration [39–41].

Conversely, group III (received exosomes only) showed the closest image to control group I with marked improvement in TBs’ number and structure in comparison to group II. There was a reduction in inflammation with intact CVP ganglion tissue.

Previous studies indicated the regenerative potential of (BM-MSC)-derived exosomes on TBs and nerve regeneration but the underlying mechanism was not fully understood. It was proved that exosomes can improve recovery of the degeneration induced by Alzheimer’s disease on CVPs’ taste buds [27]. In addition, gingival-MSC-derived exosomes were verified to facilitate TBs regeneration and reinnervation in tongue cancer patients following surgery [42].

PN regeneration following injury involves several substantial processes, including activation and transformation of SCs phenotype, development of neuronal soma, axonal regrowth, neurovascular regeneration, and regulation of inflammation [13, 43].

The article "Regenerative potentials of bone marrow mesenchymal stem cells derived exosomes or its combination with zinc in recovery of degenerated circumvallate papilla following surgical bilateral transection of glossopharyngeal nerve in rats" was retracted in 2025. Reasons: duplicated images; overlap with earlier publications; unreliable results or conclusions; concerns about the images.

It was confirmed that exosomes restrain the apoptosis of SCs and enhance their proliferation in rats. SCs perform a fundamental function in PN regeneration following injury, as they dedifferentiate into progenitor cells that undergo a phenotypic alteration. Redifferentiation occurs when newly formed axons encounter SCs and complete nerve repair [44, 45].

Recently, Adpaikar et al., 2023 revealed that a subset of differentiated CK8-positive taste receptor cells in CVP undergoes dedifferentiation, proliferation and acquires a temporary progenitor cell-like state in response to GPN transection. Later, the dedifferentiated taste cells and resident progenitor cells improve the regeneration of TBs [6]. Furthermore, Wang et al., 2019 demonstrated that MSC exosomes activate notch signaling to promote the proliferation, migration, and protein production of adult dermal fibroblasts [46]. We postulated that exosomes in the current work enhance those processes as well and accelerate the regeneration rate.

Several studies demonstrated that 28 days after spinal cord injury, BM-MSC-derived exosomes reduce apoptosis and inflammatory response. It decreases the apoptotic proteins expression levels of (Bax, cleaved caspase-3, -9), and increases the anti-apoptotic protein (Bcl-2) level. In addition, it reduces proinflammatory, elevates anti-inflammatory factors expression, and downregulates inflammatory cytokines secretion, like IL-6, TNF-α, and IFN-γ. Moreover, it promotes neurological recovery by decreasing neuronal apoptosis rate through the activation of the Wnt/β-catenin and inhibiting the TLR4/MyD88/NF-κB signaling pathways [47–49].

In spite that several previous studies demonstrated that using ZnCl_2_ as a supplement had a promising effect on neurogenesis including neuronal differentiation and axonal extension [50–52], our histological results of group IV (received exosomes + ZnCl_2_) showed negative results in comparison to group III including numerous immature TBs some of them exhibited signs of degeneration, shrunken nerve plexus with signs of ganglion cells degeneration, and inflammatory cells infiltration. Several explanations could be brought up to comprehend those results.

Several studies have discussed the promising effect of ZnCl_2_ in the treatment of different illnesses. The selected dose of ZnCl2 in the current study (5 mg/kg-IP) was used according to previously published work. Moustafa SA, 2004 study showed the antioxidant and antihyperglycemic effect of ZnCl2 (5 mg/kg-IP) in the retina and pancreas of diabetic rats [25]. Furthermore, Li et al., 2022 stated that ZnCl_2_ (10 mg/kg-IP) significantly recovers neurological function following cerebral ischemia by promoting astrocyte-induced angiogenesis in rats. Additionally, Johnson et al., 2011 calculated the maximum tolerated dose (MTD) of ZnCl_2_ and it was set at 60.00 mg/kg/day in rats [53, 54].

The article "Regenerative potentials of bone marrow mesenchymal stem cells derived exosomes or its combination with zinc in recovery of degenerated circumvallate papilla following surgical bilateral transection of glossopharyngeal nerve in rats" was retracted in 2025. Reasons: duplicated images; overlap with earlier publications; unreliable results or conclusions; concerns about the images.

Zn^2+^ was expected to be involved in neuronal damage after nerve injury, it was proven that impairment of Zn^2+^ homeostasis (as in traumatic brain injury) results in the subsequent increase of the postsynaptic cellular Zn^2+^ level and leads to a powerful neurotoxic effect [55]. Li et al., 2017 showed that Zn^2+^ level elevated quickly in the retinal ganglion cells following optic nerve injury, which limits the regenerative capability of the optic nerve. They found that chelating Zn^2+^ improved ganglion cell survival and considerable axon regeneration [56].

In other perspectives, high concentrations of free Zn^2+^ are stored by neurons in their presynaptic terminals, where they are released during depolarization. In the case of trauma or injured nerve, presynaptic boutons lose Zn^2+^, which then accumulates in damaged neurons [57]. When the Zn^2+^ homeostatic system becomes inefficient, the elevated intracellular Zn^2+^ levels trigger several cellular signaling pathways that cause cell death and atrophy [55, 58]. Moreover, accumulation of intracellular Zn^2+^ (from exogenous or intracellular sources), made it act as a neurotoxin by activating molecules that promote apoptosis, such as potassium channels and p38 [57].

It was documented that Zn^2+^ affects signaling within taste cells when it is released in response to taste stimuli. It was also found that taste cells type II and III expressed zinc transporter which is responsible for Zn^2+^ loading into synaptic vesicles [59]. The released Zn^2+^ is targeted at the postsynaptic terminal by the ionotropic glutamate N-methyl-D-aspartate receptors which is expressed at the basal part of TBs.

Likewise, it was proved that the extracellular application of ZnCl_2_ inhibits the transient receptor potential melastatin 5 channel activity, which is expressed by taste cells and is believed to be implicated in membrane potential coordination [60].

Furthermore, Zn^2+^ was found to be a potent inhibitor of sweetness and bitterness which is detected by T1R1/T1R3 receptors in type II cells with more than 70% reduction in taste. Thus, it could be concluded that Zn^2+^ accumulation may be attributed to cell damage of taste cells with subsequent effects on taste perception [61].

Notch signaling plays an important role in taste decisions by determining type II and type III cell fates in embryonic and adult TBs cell lineage [62, 63]. Baek et al., 2007 have demonstrated the suppression and reduction of notch signaling by Zn^2+^ via the PI3K–Akt signaling pathway [64]. This may explain the increased number of immature TBs within the gustatory epithelium in group IV.

The article "Regenerative potentials of bone marrow mesenchymal stem cells derived exosomes or its combination with zinc in recovery of degenerated circumvallate papilla following surgical bilateral transection of glossopharyngeal nerve in rats" was retracted in 2025. Reasons: duplicated images; overlap with earlier publications; unreliable results or conclusions; concerns about the images.

Interestingly, the RT-PCR and biochemical analysis of the ongoing study correlated with histopathological and histomorphometric results. In the present study, CK8 protein exhibited higher statistical significance values in group III in comparison to other experimental groups, while group II exhibited the lowest value. CK8 is a marker of fully differentiated taste receptor cells of CVP in rats and disappears in degenerated taste cells [6, 65]. Furthermore, a negative expression of antibodies against CK8 in denervated CVP was reported [66].

The lower values in group IV denote that the number of differentiated taste cells was markedly lesser than in group III. This indicates a reinnervation process and recovery in response to (BM-MSC)-derived exosomes treatment which affected negatively in case of combination with Zn^2+^.

The statistical results of BDNF expression in the present research revealed that group III was higher than all other experimental groups, while group II was the lowest. BDNF is expressed in TB cells and is required for its innervation and development. BDNF deficiency is linked to papillae malformation, altered innervation and taste discrimination [67, 68]. It was reported that 4 weeks following denervation, only a few TBs expressed BDNF [37] This denotes the accelerated regeneration of TBs in groups III and IV in comparison to group II in the present study. Zn^2+^ supplementation has been implicated in the signaling regulation of BDNF and increased its expression in mice models [69, 70]. The relatively high values in group IV may be attributed to the increased number of immature TBs, this suggests that higher values of BDNF are not enough to ensure actual recovery.

The biochemical analysis of the present study tested GSH and MDA as antioxidant and oxidative stress markers respectively, for assessment of degree of nerve regeneration and damage. Nerve tissue repair depends on many factors and involves different mechanisms, oxidative stress is one of them [71].

GSH is an important antioxidant in the body in nearly every organ. Multiple studies highlighted its role in the preservation of intracellular redox homeostasis, repair, and the cellular defense cascade against oxidative injury [72, 73]. MDA is one of the final peroxidation products in the cells, its level increases in response to elevated free radicals’ production. It has been employed as a biomarker to assess oxidative stress in a variety of illnesses, such as neurological disorders and cancer [74, 75].

The article "Regenerative potentials of bone marrow mesenchymal stem cells derived exosomes or its combination with zinc in recovery of degenerated circumvallate papilla following surgical bilateral transection of glossopharyngeal nerve in rats" was retracted in 2025. Reasons: duplicated images; overlap with earlier publications; unreliable results or conclusions; concerns about the images.

Regarding GSH, the results of groups I and III were significantly higher than groups II and IV by more than twice. On the contrary, MDA was significantly higher in groups II & IV when compared with groups I and III. These signifies that the results of group III were markedly superior to group IV with increased levels of antioxidants and decreased levels of oxidative stresses. It was proven that higher amounts of reactive oxygen species in neurons are linked to Zn^2+^ -induced cell death [57]. Furthermore, a previous study verified that the concentrations of GSH were significantly decreased whereas the MDA was significantly increased in the brain of rats who exposed to zinc oxide nanoparticles injection [75].

## Conclusions

Taste buds are neuroepithelial cells, that have unique features in between epithelial and nervous tissues, and their presence is dependent on normal nerve supply. The present work has proven that BM-MSC-derived exosomes accelerated the regeneration process of GPN after surgical cutting with subsequent improvement of taste buds and ganglion. The combination of exosomes with ZnCl_2_ was expected to enhance its regenerative power. However, the current results provide evidence that ZnCl_2_ did not reach the expectancy with little improvement when compared to the group that received no treatment. This adverse effect is believed to be related essentially to the consequence of nerve transection with subsequent imbalance in Ca^2+^ and Zn^2+^ ions hemostasis. Our hypothesis suggests that the external dose of ZnCl_2_ causes a negative effect that interferes with exosomes function. We recommend that the maximum safe dose of ZnCl_2_ in rats needs to be reinvestigated to ensure that the damage is not related to an inaccurate dose. In addition, future studies should focus on investigating the analytical or pharmacological properties of ZnCl_2_ when combined with exosomes. These results highlight the need to establish limitations on Zn^2+^ supplementations and extra use in other oral hygiene products. Extra care should be given after oral surgeries that involve nerve injury.

## Electronic supplementary material

Below is the link to the electronic supplementary material.

Supplementary Material 1

Supplementary Material 2

## Data Availability

All data supporting the findings of this study are available within the paper and its supplementary information.

## Abbreviations

CVP: Circumvallate papillae
GPN: Glossopharyngeal nerve
TBs: Taste buds
PN: Peripheral nerve
BM-MSC: Bone marrow mesenchymal stem cells derived exosomes
Zn2+: Zinc
IACUC: Institutional Animal Care and Use Committee
IP: Intraperitoneal
IV: Intravenous
ZnCl2: Zinc chloride
H&E: Hematoxylin and Eosin
RT-PCR: Reverse transcription polymerase chain reaction
CK8: Cytokeratin 8
PBS: Phosphate-buffered saline
ELISA: Enzyme Linked Immunosorbent Assay
BDNF: Brain-derived neurotrophic factor
MDA: Malondialdehyde
GSH: Reduced glutathione
CI: Confidence intervals
SD: Standard deviation
CT: Connective Tissue
SCs: Schwann cells
